The article "Hybrid Sharpening Transformation Approach for Multifocus Image Fusion Using Medical and Nonmedical Images" was published in 2021. Journal: J Healthc Eng.

# Hybrid Sharpening Transformation Approach for Multifocus Image Fusion Using Medical and Nonmedical Images

**DOI:** 10.1155/2021/7000991

**Published:** 2021-12-11

**Authors:** Sarwar Shah Khan, Muzammil Khan, Yasser Alharbi, Usman Haider, Kifayat Ullah, Shahab Haider

**Affiliations:** ^1^Department of Software Engineering, University of Sialkot, Sialkot 51310, Pakistan; ^2^Department of Computer & Software Technology, University of Swat, Swat 19130, Pakistan; ^3^College of Computer Science & Engineering, University of Hail, Ha'il, Saudi Arabia; ^4^Ghulam Ishaq Khan Institute of Engineering Science and Technology, Topi Swabi, Pakistan; ^5^Department of Computer Science, City University of Science and IT, Peshawar, Pakistan

## Abstract

In this study, we introduced a preprocessing novel transformation approach for multifocus image fusion. In the multifocus image, fusion has generated a high informative image by merging two source images with different areas or objects in focus. Acutely the preprocessing means sharpening performed on the images before applying fusion techniques. In this paper, along with the novel concept, a new sharpening technique, Laplacian filter + discrete Fourier transform (LF + DFT), is also proposed. The LF is used to recognize the meaningful discontinuities in an image. DFT recognizes that the rapid change in the image is like sudden changes in the frequencies, low-frequency to high-frequency in the images. The aim of image sharpening is to highlight the key features, identifying the minor details, and sharpen the edges while the previous methods are not so effective. To validate the effectiveness the proposed method, the fusion is performed by a couple of advanced techniques such as stationary wavelet transform (SWT) and discrete wavelet transform (DWT) with both types of images like grayscale and color image. The experiments are performed on nonmedical and medical (breast medical CT and MRI images) datasets. The experimental results demonstrate that the proposed method outperforms all evaluated qualitative and quantitative metrics. Quantitative assessment is performed by eight well-known metrics, and every metric described its own feature by which it is easily assumed that the proposed method is superior. The experimental results of the proposed technique SWT (LF + DFT) are summarized for evaluation matrices such as RMSE (5.6761), PFE (3.4378), MAE (0.4010), entropy (9.0121), SNR (26.8609), PSNR (40.1349), CC (0.9978), and ERGAS (2.2589) using clock dataset.

## 1. Introduction

In the field of image fusion, the subfield multifocus image fusion is one of the most significant and valuable approaches to handle the problem of defocusing that some parts of the image are not in focus and blurred due to the limited depth of focus in the optical lens of traditional cameras or large aperture and microscopes cameras. In multifocus image fusion, various images of a similar scene but with different focus settings can be merged into a signal image (one image) with more information, where all the parts of the image are entirely focused. The practical technique of multifocus image fusion should need to accomplish the requirements that all the information of the focused regions in the source images is preserved in the resultant image [1]. Due to this, the resulting image is well-informative and complete. Multifocus image fusion is applicable in a wide range of applications such as environmental monitoring, image analysis [2], military technology, medical imaging [3], remote sensing, hyperspectral image analysis [4], computer vision, object recognition [5], and image deblurring [6].

The article "Hybrid Sharpening Transformation Approach for Multifocus Image Fusion Using Medical and Nonmedical Images" was published in 2021. Journal: J Healthc Eng.

In the multifocus image, fusion has been introduced as a large number of techniques over the past couple of decades; some of them are very popular methods and achieve high accuracy, such as stationary wavelet transform (SWT) [7], discrete wavelet transform (DWT), dual-tree complex wavelet transform (DT-CWT), and discrete cosine transform (DCT) [2]. Most multifocus image fusion techniques are divided into four major classes [1, 8]. The first category is multiscale decomposition or frequency domain techniques such as wavelet transformation [8, 9], complex wavelet transformation [1, 10], nonsubsampled contourlet transform [11], DWT [2], and SWT [12]. The second category is sparse representation techniques like an adaptive SR model proposed in [13] for simultaneous image fusion and denoising and multitask sparse representation technique [14]. The third category of techniques is based on computational photography, such as light-field rendering [15]. This kind of technique finds more of the physical formation of multifocus images and reconstructs the all-in-focus images. The last category of techniques performed in the spatial domain, which can make full use of the spatial context and provide spatial consistency or spatial domain, includes averaging [2, 16], minimum [2,17], intensity hue saturation (IHS) [2,18], principal component analysis (PCA) [2,19], and Gram–Schmidt [20] techniques.

In this paper, a new concept has been proposed in the image fusion environment for multifocus image fusion. The key contributions of this work are summarized as follows:

- The new concept is that image enhancement or image sharpening techniques are used before image fusion; in other words, the preprocessed step is performed before applying image fusion techniques.
- The preprocessed step is beneficial before the image fusion because the sharpening methods are helpful for recognizing the meaningful discontinuities in an image, i.e., edges information or edges detection.
- All the standard techniques of image fusion have directly fused the images and generated the resultant image. In this work, first, the source images were enhanced, using the proposed hybrid enhancement method such as LF + DFT (Laplacian filter + discrete Fourier transform) and other popular enhancement methods (Laplacian filter (LF) and unsharp masking (UM)).
- Second, the enhanced images were fused by popular fusion methods such as DWT, SWT, and generated more informative and meaningful resultant images as demonstrated in Figure 1. The performance of the novel proposed method is outperformed as compared with the state-of-art methods.

The article "Hybrid Sharpening Transformation Approach for Multifocus Image Fusion Using Medical and Nonmedical Images" was published in 2021. Journal: J Healthc Eng.

The rest of the paper is organized as follows.  Section 2 briefly describes the related work of multifocus image fusion.  Section 3 describes the proposed methodology, such as Laplacian filter + discrete Fourier transform with DWT and SWT.  Section 4 shortly describes the performance measures.  Section 5 gives the experimental results and discussion, and the paper is concluded in Section 6.

## 2. Literature Study

Multifocus image fusion is one of the most significant areas of image processing, and a lot of advanced techniques have been proposed in a couple of decades. Several works have been carried out in the spatial domain. Principal component analysis (PCA) is the most frequently used method and is specially designed to generate visible results regarded as sharp edges and highly preserved spatial characteristics [21]. The intensity hue saturation (IHS) technique effectively transforms the image from red, green, and blue (RGB) domain into spatial (I) and spectral (H, S) information [22]. The PCA and IHS have one significant advantage: both can use an arbitrary number of channels [23]. Brovey technique is mathematical formulas of the Brovey transform (BT), introduced by American scientist Bob Brovey. BT is different sources that capture a simple technique for merging the information. Brovey is also called the color normalization transform (CNT) because it involves a red, green, blue (RGB) color transform approach [24]. Average and maximum/minimum selection is also spatial-domain method [25]. Many spatial-domain methods are complicated and time-consuming, and these techniques produce poor results because they usually produce spectral distortions in the fused images, and the produced image is of low contrast, which contains less information comparatively.

Image fusion is also based on frequency domain techniques such as discrete cosine transform (DCT), the frequency information (pixels) is very effective in obtaining the details and outlines of an image, and DCT is the proper working mechanism with frequencies. It provides a fast and noncomplex solution because it uses only cosine components for the transformation. The IDCT reconstructs the original pixel values from the frequencies acquired from DCT [26]. The discrete cosine harmonic wavelet transform (DC-HWT) is the advanced version of DCT. In DC-HWT, the signal is decomposed by grouping the DCT coefficients similarly to DFT coefficients except for the conjugate operations in laying the coefficients symmetrical (accurate as DCT).

The article "Hybrid Sharpening Transformation Approach for Multifocus Image Fusion Using Medical and Nonmedical Images" was published in 2021. Journal: J Healthc Eng.

Further, symmetric placement is also not significant due to the definition of DCT [27]. These groups' inverse DCT (IDCT) results in discrete cosine harmonic wavelet coefficients (DC-HWCs). The DCT of these processed sub-bands (DC-HWCs) results in sub-band DCT coefficients, which are repositioned in their corresponding positions to retrieve the overall DCT spectrum at the original sampling rate. Details of DC-HWT are provided in reference [28]. The dual-tree complex wavelet transform (DT-CWT) is based on a couple of parallel trees, the first one represents the odd samples, and the second one represents the actual samples generated at the first level. The parallel trees render the signal delays necessary for each level and, therefore, eradicate aliasing effects and attain shift-invariance [29]. Discrete wavelet transform (DWT) is the mathematical tool introduced in the 1980s, and it is an instrumental technique for image fusion in the wavelet transformation process [1] but with the following drawbacks: it retains the vertical and horizontal features only, it is lack of shifting invariance, it suffers through ringing artifacts and reduces the quality of the resultant fused image, it is lack of shifting dimensionality, and it is not suitable for edge places due to missing edges during the process. The technique DWT is not a time-invariant transformation technique, which means that “with periodic signal extension, the DWT of a translated version of a signal *X* is not, in general, the translated version of the DWT of *X*.”

The stationary wavelet transform (SWT) is a wavelet transform developed to overcome the deficiency of translation invariance of the DWT. The SWT is an entire shift-invariant transform, which up-samples the filters by putting zeros among the filter coefficients to overcome the down-sampling step of the decimated approach [2]. They provide improved time-frequency localization, and the design is simple. Appropriate high-pass and low-pass filters have used the data at each level, producing two sequences at the next level. In the decimated approach, the filters are applied for the rows at first and then for the columns [7, 30]. The SWT filter bank structure is given in Figure 2.

The article "Hybrid Sharpening Transformation Approach for Multifocus Image Fusion Using Medical and Nonmedical Images" was published in 2021. Journal: J Healthc Eng.

The images are broken down into horizontal and vertical approximations by employing column-wise and row-wise low-pass and high-pass filters [31]. The same filtration decomposes elements row-wise and column-wise to acquire vertical, horizontal, and diagonal approximation. The low-pass and high-pass filters preserve the low and high frequencies and provide detailed information at respective frequencies.

## 3. Proposed Methodology

In this article, the novel idea is proposed, which is the first time involved in multifocus image fusion to increase the accuracy (the visibility of objects). The novel concept is preprocessed evaluation of images before fusion. The fusion is performed by the two standard methods such as DWT and SWT to validate the proposed techniques. The complete process is demonstrated in Figure 3, and the proposed techniques are elaborated as follows.

### 3.1. Laplacian Filter (LF)

The Laplacian filter of an image highlights an area of rapid intensity change. Hence, the LF is used for the edge-sharpening [27, 30, 32]. This operator is exceptionally well at identifying the critical information in an image. Any feature with sharp discontinuity will be sharpening by an LF. Laplacian operator is also known as a derivative operator, used to identify an image's key features. The critical difference between the Laplacian filter and other filters such as Prewitt, Roberts, Kirsch, Robinson, and Sobel [27, 33] is that all these filters use first-order derivative masks, but LF is a second-order derivative mask. LF sharpens the “Knee MRI medical image,” which demonstrates the difference between source and LF sharpen images. The Laplacian equation is as follows:

(1) $$\begin{array}{c} \Delta^{2}I=\left(\frac{\partial^{2}G}{\partial x^{2}}+\frac{\partial^{2}G}{\partial y^{2}}\right)⊗I\left(x,y\right). \end{array}$$

### 3.2. Unsharp Mask (UM)

An “unsharp mask” is a simple sharpen image operator, contrary to what its name might lead you to believe. However, actually, the name is derived from the fact that it sharpens edges through a process that deducts an unsharp version of a picture from the reference picture and detects the presence of edges, making the unsharp mask (effective a high-pass filter) [19]. Sharpening can demonstrate the texture and detail of the image. This is probably the common type of sharpening and can be executed with nearly any image. The unsharp mask cannot add artifacts or additional detail in the image, but it can highly enhance the appearance by increasing small-scale acutance [33, 34] and making important details easier to identify. The unsharp mask method is usually used in the photographic and printing industry applications for crispening edges. In sharpening images, the image size does not change, and it remains similar, but an unsharp mask improves the sharpness of an image by increasing the acutance only. In the unsharp masking technique, the sharper image *a*(*x*, *y*) will be produced from the input image *b*(*x*, *y*) as

(2) $$\begin{array}{c} a\left(x,y\right)=b\left(x,y\right)+\lambda c\left(x,y\right), \end{array}$$

where *c* (*x*, *y*) is the correction signal calculated as the output of a high-pass filter and *λ* is a positive scaling factor that controls the level of contrast sweetening achieved at the output [32,35]. Unsharp masking sharpens the “Knee MRI medical image,” demonstrating the difference between source, LF, and unsharp masking sharpen images.

The article "Hybrid Sharpening Transformation Approach for Multifocus Image Fusion Using Medical and Nonmedical Images" was published in 2021. Journal: J Healthc Eng.

### 3.3. LF + DFT Method

The hybrid sharpening technique (LF + DFT) is proposed in this study for multifocus image fusion. The hybrid approach is the merger of the advantages of LF and DFT methods. The LF is used to recognize the meaningful discontinuities in an image, i.e., edges information or edges detection. In other words, LF is a derivative operator used to find the region of rapid change in the picture. The rapid change in the image is like sudden changes in the frequencies, low-frequency to high-frequency [36]. The DFT is a common approach used to compute the frequency information as discrete. The frequency information is considered an important way in the picture enhancement [33, 37]. Therefore, to make a beneficial way of sharpening, the frequency information of Fourier transform is combined with the second derivative masking of Laplacian filter in the novel technique. Here is the involvement of spatial conversion to the frequency and inverse (see equations (4) and (5)). So, this is the reason for calling that the cross-domain method.

For a two-dimensional square image with *N* × *N*, the DFT equation is given as follows:

(3) $$\begin{array}{c} F\left(x,y\right)=\sum_{m=0}^{M-1}\sum_{n=0}^{N-1}f\left(m,n\right)e^{-y2\pi \left(xm/N+yn/N\right)}, \end{array}$$

where *f*(*m*, *n*) is the spatial-domain image, and the exponential term is the basis operation representing every point *F*(*x*, *y*) in the Fourier space. The formulation can be construed as follows: the value of every point *F*(*x*, *y*) is acquired by multiplying the spatial image with the representing base operation and summing the results.

The primary operations are cosine and sine waves with growing frequencies, i.e., *F*(*0*, *0*) presents the DC components of the image which corresponds to the average brightness and *F*(*N* − 1, *N* − 1) presents the highest frequency.

The article "Hybrid Sharpening Transformation Approach for Multifocus Image Fusion Using Medical and Nonmedical Images" was published in 2021. Journal: J Healthc Eng.

Similarly, the frequency domain image can be retranslated (inverse transform) to the spatial domain, shown in Figure 4. The inverse frequency transform is as follows:

(4) $$\begin{array}{c} f\left(a,b\right)=\frac{1}{N^{2}}\sum_{k=0}^{M-1}\sum_{l=0}^{N-1}F\left(k,l\right)e^{l2\pi \left(ka/N+lb/N\right)}. \end{array}$$

In the proposed technique, for a two-dimensional square image with *N* × *N* resolution, the Laplacian equation (2) and Fourier equation (4) are given:

(5) $$\begin{array}{c} L\left(\Delta \right)=\sum_{a=0}^{M-1}\sum_{b=0}^{N-1}\left(\Delta^{2}I\right)e^{-l2\pi \left(km/N+\ln/N\right)}. \end{array}$$

The apparent sharpness of an image is increased, which is the combination of two factors, i.e., resolution and acutance. Resolution is straightforward and not subjective, which means the size of the image file in terms of the number of pixels. With all other factors remaining equal, the higher the resolution of the image is—the more pixels it has—the sharper it can be. Acutance, a measure of the contrast at an edge, is subjective and a little complicated comparatively. There is no unit for acutance—you either think an edge has contrast or think it does not. Edges that have more contrast appear to have a more defined edge to the human visual system. LF + DFT sharpens the “Knee MRI medical image,” which demonstrates the difference between source, LF, unsharp masking, and sharpen images in Figure 5.

## 4. Performance Metrics

The quantitative evaluation aims to identify the performance of the proposed methods and existing methods on various measures, and every measure has its properties.  Table 1 briefly describes the well-known statistical metrics.

## 5. Experimentation

### 5.1. Datasets

In this letter, the experimentations are performed on four image sets; two are grayscale image sets including “Clocks” and “Books,” and the other two are color image sets such as “Toys” and “Building and card.” The grayscale image sets are provided by authors, and the color image sets are acquired from “Lytro multifocus datasets” [43]. These image sets are used for testing multifocus images for the experimental evaluation of novel techniques. The size of the grayscale image sets (test images) is 512 × 512, and the size of the color image sets is 520 × 520 pixels.

### 5.2. Experimental Results and Discussion

In this section, the experimentation is conducted on different multifocus image sets for the proposed hybrid methods. The proposed hybrid methods like DWT + LF, DWT + unsharp masking, DWT + (LF + DFT), SWT + LF, SWT + unsharp masking, and SWT + (LF + DFT) are compared with the traditional methods such as average method (spatial-domain methods), minimum method, DWT (frequency domain method), and SWT methods. The algorithms are implemented, and the simulations are performed using the MATLAB 2016b application software tool. The resultant images are evaluated in two ways, i.e., quantitatively and qualitatively. For quantitative evaluation, eight well-known performance matrices, i.e., percentage fit error (PFE), entropy (E), correlation coefficient (CORR), peak signal to noise ratio (PSNR), relative dimensionless global error (ERGAS), mean absolute error (MAE), signal to noise ratio (SNR), and root mean square error (RMSE) are used to measure the performance of resultant images of old and new methods. The quantitative results of the new approaches are improved for the “Clocks,” “Books,” “Toys,” “Building and card,” and “Breast Medical (CT and MRI images)” image sets, as shown in Tables 2–6. All the performance metrics show better results for the proposed approaches on all image sets, which show the capability of the new approaches in fusion environment.

The article "Hybrid Sharpening Transformation Approach for Multifocus Image Fusion Using Medical and Nonmedical Images" was published in 2021. Journal: J Healthc Eng.

RMSE indicates the difference between the true image and the resultant image. The smallest values show excellent results. PFE is computing the norm of the difference among the corresponding pixels of the true and resultant image to the norm of the true image. The low values indicate superior results. MAE is the absolute error to calculate and validate the difference between resultant and reference images. Here, MAE values are small for the proposed methods on both image sets, promising results. The large value of entropy expresses the good results; hence, for the “Books” image set, the DWT technique has a large value, while the “Clock” image sets the proposed methods to demonstrate the impressive results. The CORR is a quantitative measure that demonstrates the correlation between the true image and the resultant image. When the true and resultant images are similar, the value will be near to one. PSNR is specifically used for the measurement of spatial quality in the image. SNR is the performance measure used to find the ratio among information and noise of the resultant image. ERGAS is used to calculate the quality of the resultant image in terms of normalization average error of each channel of the processed image. The quantitative results of the proposed methods are well performed as compared with traditional methods. According to the results shown in Figures 6–10, the SWT + (LF + DFT) method is superior among all proposed methods.

The qualitative analysis is a significant evaluation metric in multifocus image fusion. The scientists performed fusion on simple multifocus images. All the fusion methods are directly employed to the multifocus images and improved the results. However, in this article, the new concept is introduced as a preprocessing step before fusion. This concept is firstly proposed in fusion environment. The preprocessed step is involved in sharpening the images. Three image sharpening techniques are used as a preprocessed step like Laplacian filter, unsharp masking, and LF + DFT. From Figures 11–15, (a) and (b) both are source images, while (c) and (d) are sharpen images by Laplacian filter, (e) and (f) are sharpen images by unsharp masking, and (g) and (h) are sharpen images by LF + DFT for “Clocks,” “Books,” “Toys,” and “Building and Cards” image sets, respectively.

The article "Hybrid Sharpening Transformation Approach for Multifocus Image Fusion Using Medical and Nonmedical Images" was published in 2021. Journal: J Healthc Eng.

## 6. Conclusions

In this paper, we are mainly trying to solve the problem of the out-of-focus blur part of an image. To achieve this goal, we introduced a new concept of sharpening the edges or enhancing the image before fusing the multifocus source images. Laplacian filter does the preprocessing step (sharpen the edges), unsharp masking, and newly proposed Laplacian filter + discrete Fourier transform (LF + DFT) sharpen method. The sharpening concept is firstly proposed in a fusion environment, and the experimental results demonstrate the superiority of the new concept. After sharpening the images, fusion is performed by stationary wavelet transform (SWT) and discrete wavelet transform (DWT) techniques. The experiments are conducted on color and grayscale datasets to validate the effectualness of the proposed technique. Four datasets “Clock,” “Book,” “Toy,” “Building and Card,” and “Breast Medical CT and MRI images” are used for experimentation The proposed technique is evaluated visually and statistically, and for statistical assessment, we used eight well-known metrics such as percentage fit error, entropy, correlation coefficient, peak signal to noise ratio, relative dimensionless global error, mean absolute error, signal to noise ratio, and root mean square error which indicates that the new method outperformed among all state-of-the-art methods. In this work, one major future challenge is that the proposed scheme is not time efficient because of the preprocessed step before image fusion compared with simple fusion methods.

## Figures and Tables

**Figure 1:** Systematic approach for multifocus image fusion.

**Figure 2:** SWT filter bank structure.

**Figure 3:** The abstract flow-chart of the proposed scheme.

**Figure 4:** Framework of the proposed approach.

**Figure 5:** The sharpen results of “Knee MRI medical image”: (a) source image, (b) sharpen image by Laplacian filter, (c) sharpen image by unsharp masking, and (d) LF + DFT sharpen image.

The article "Hybrid Sharpening Transformation Approach for Multifocus Image Fusion Using Medical and Nonmedical Images" was published in 2021. Journal: J Healthc Eng.

**Figure 6:** The fusion results of “clocks image set”: (a) average fused, (b) minimum fused, (c) DWT fused, (d) SWT fused, (e) DWT + LF fused, (f) DWT + UM, (g) DWT + (LF + DFT), (h) SWT + LF, (i) SWT + UM, and (j) SWT + (LF + DFT).

**Figure 7:** The fusion results of “books image set”: (a) average fused, (b) minimum fused, (c) DWT fused, (d) SWT fused, (e) DWT + LF fused, (f) DWT + UM, (g) DWT + (LF + DFT), (h) SWT + LF, (i) SWT + UM, and (j) SWT + (LF + DFT).

**Figure 8:** The fusion results of “toys image set”: (a) average fused, (b) minimum fused, (c) DWT fused, (d) SWT fused, (e) DWT + LF fused, (f) DWT + UM, (g) DWT + (LF + DFT), (h) SWT + LF, (i) SWT + UM, and (j) SWT + (LF + DFT).

**Figure 9:** The fusion results of “building and card image set”: (a) average fused, (b) minimum fused, (c) DWT fused, (d) SWT fused, (e) DWT + LF fused, (f) DWT + UM, (g) DWT + (LF + DFT), (h) SWT + LF, (i) SWT + UM, and (j) SWT + (LF + DFT).

**Figure 10:** The fusion results of “medical images”: (a) average fused, (b) minimum fused, (c) DWT fused, (d) SWT fused, (e) DWT + LF fused, (f) DWT + UM, (g) DWT + (LF + DFT), (h) SWT + LF, (i) SWT + UM, and (j) SWT + (LF + DFT).

**Figure 11:** The sharpen results of “clocks image set”: (a, b) two source images, (c, d) sharpen images by Laplacian filter, (e, f) sharpened images by unsharp masking, and (g, h) LF + DFT sharpen images.

**Figure 12:** The sharpen results of “books image set”: (a, b) two source images, (c, d) sharpen images by Laplacian filter, (e, f) sharpened images by unsharp masking, and (g, h) LF + DFT sharpen images.

**Figure 13:** The sharpen results of “toys image set”: (a, b) two source images, (c, d) sharpen images by Laplacian filter, (e, f) sharpened images by unsharp masking, and (g, h) LF + DFT sharpen images.

**Figure 14:** The sharpen results of “building and card image set”: (a, b) two source images, (c, d) sharpen images by Laplacian filter, (e, f) sharpened images by unsharp masking, and (g, h) LF + DFT sharpen images.

**Figure 15:** The sharpen results of “medical images” (a, b) two CT and MRI medical images, (c, d) sharpen images by Laplacian filter, (e, f) sharpened images by unsharp masking, and (g, h) LF + DF\T sharpen images.

**Table 1:** Measurements to evaluate the experimental results.

Quality metrics	Description	Formula	What value to look for best fusion	Reference
RMSE	The RMSE is generally used to calculate the difference among the true image and resultant image by directly calculating the variations in pixel values. RMSE is highly indicating the spectral quality of the resultant image.	$\text{RMSE}=\sqrt{1/MN\sum_{a=1}^{M}\sum_{b=1}^{N}{\left(I_{z}\left(a,b\right)-I_{f}\left(a,b\right)\right)}^{2}}$	Lower (close to zero)	[38]

PFE	It is calculated as the norm of the difference among the corresponding pixels of the true image and resultant image to the norm of the true image.	PFE=[norm(*I*_*z*_ − *I*_*f*_)/norm(*I*_*z*_)+norm(*I*_*z*_ − *I*_*f*_)/norm(*I*_*f*_)] × 100	Lower (equal to zero)	[2]

MAE	It gives the MAE of the corresponding pixels in the true image and resultant image.	$\begin{array}{c} \text{MAE}=1/MN\sum_{a=1}^{M}\sum_{b=1}^{N}\left|I_{z}\left(a,b\right)-I_{p}\left(a,b\right)\right|+\\ 1/MN\sum_{a=1}^{M}\sum_{b=1}^{N}\left|I_{x}\left(a,b\right)-I_{p}\left(a,b\right)\right| \end{array}$	Lower (equal to zero)	[2]

Entropy	Entropy (*E*) is a significant quantitative metric, which can be used to distinguish the texture, appearance, or information contents in the image.	*E*=−∑_*k*=0_^*G*−1^*S*_*k*_log *S*_*k*_	Higher value	[18]

SNR	SNR is the performance measure used to find the ratio among information and noise of the resultant image.	SNR=10 log_10_(∑_*a*=1_^*M*^∑_*b*=1_^*N*^(*I*_*z*_(*a*, *b*))^2^/∑_*a*=1_^*M*^∑_*b*=1_^*N*^(*I*_*z*_(*a*, *b*) − *I*_*p*_(*a*, *b*))^2^)	Higher value	[39]

PSNR	PSNR is one of the significant metrics and most commonly used in fusion. PSNR is specifically used for the measurement of spatial quality in the image. The computation is performed by the value of grey levels divided by the identical pixels in the true and the resultant images.	PSNR=20 log[*G*^2^/1/*M* × *N*∑_*a*=1_^*M*^∑_*b*=1_^*N*^(*I*_*z*_(*a*, *b*) − *I*_*p*_(*a*, *b*))^2^]	Higher value	[40]

CC	The CORR is a quantitative metric that demonstrates the correlation among the true image and the resultant image. When the true and resultant images look the same, the value will be near to one. If the true and resultant images are dissimilar, then the value will be near zero.	$\begin{array}{c} \text{Corr}=2C_{zp}/C_{z}+C_{P}\\ C_{zp}=\sum_{a=1}^{M}\sum_{b=1}^{N}I_{z}\left(a,b\right)*I_{p}\left(a,b\right)\\ C_{z}=\sum_{a=1}^{M}\sum_{b=1}^{N}I_{z}{\left(a,b\right)}^{2}\\ C_{p}=\sum_{a=1}^{M}\sum_{b=1}^{N}I_{p}{\left(a,b\right)}^{2} \end{array}$	Higher value (close to +1)	[30, 41]

ERGAS	ERGAS is used to calculate the quality of the resultant image in terms of the normalization average error of each channel (band) of the processed image.	ERGAS=100d*a*/d*b*[1/*n*∑_*i*=1_^*n*^(RMSE^2^/mean^2^)]^1/2^	Lower (equal to zero)	[42]

The article "Hybrid Sharpening Transformation Approach for Multifocus Image Fusion Using Medical and Nonmedical Images" was published in 2021. Journal: J Healthc Eng.

**Table 2:** Statistical comparisons of multifocus image fusion on the “clocks image set.”

Methods	RMSE	PFE	MAE	Entropy	SNR	PSNR	CC	ERGAS
Average method	28.4166	23.8202	7.8278	1.9823	14.5830	35.5127	0.9144	5.7748
Minimum method	11.5217	10.5229	4.4813	4.8810	18.6569	37.5496	0.9942	4.3994
DWT	7.7077	7.0396	0.4880	7.8322	22.1487	39.2955	0.9976	2.9858
SWT	7.5158	6.8643	0.4835	8.3824	22.3677	39.4050	0.9975	2.9862
DWT (Laplacian) proposed	6.9276	3.8344	0.4174	8.6432	24.5875	39.5099	0.9979	2.9839
DWT (unsharp) proposed	7.5207	4.4390	0.4166	8.6343	24.6678	39.5500	0.9976	2.9624
DWT (LF + DFT) proposed	6.1766	3.5184	0.4107	9.0001	26.7923	40.1006	**0.9980**	2.2845
SWT (Laplacian) proposed	6.9978	3.9638	0.4110	8.8432	25.0712	39.7517	0.9978	2.8676
SWT (unsharp) proposed	6.9049	3.9811	0.4101	8.7321	25.1449	39.7886	0.9975	2.8731
SWT (LF + DFT) proposed	**5.6761**	**3.4278**	**0.4010**	**9.0121**	**26.8609**	**40.1349**	0.9978	**2.2589**

**Table 3:** Statistical comparisons of multifocus image fusion on “books image set.”

Methods	RMSE	PFE	MAE	Entropy	SNR	PSNR	CC	ERGAS
Average method	26.2368	25.2586	10.6240	7.9872	11.2489	33.9757	0.9024	10.0925
Minimum method	14.4007	13.8638	4.7984	12.3321	16.4595	36.5810	0.9900	6.7961
DWT	10.9863	10.5767	0.1636	17.2384	18.8102	37.7563	0.9944	3.2366
SWT	10.9503	10.5421	0.1635	18.0932	18.8386	37.7705	0.9945	3.2408
DWT (Laplacian) proposed	10.0025	8.9378	0.1703	18.7548	18.8151	37.8540	0.9921	2.8606
DWT (unsharp) proposed	10.7051	8.6659	0.1707	18.7384	18.7955	37.8190	0.9926	2.7746
DWT (LF + DFT) proposed	9.1990	8.7186	0.1636	21.3843	18.8614	**39.5801**	0.9964	2.4083
SWT (Laplacian) proposed	10.4319	8.3976	0.1604	18.6342	18.8665	37.8797	0.9933	2.7049
SWT (unsharp) proposed	10.4895	**8.1775**	0.1708	18.7832	18.8558	37.7342	0.9936	2.6349
SWT (LF + DFT) proposed	**9.0836**	8.2106	**0.1633**	**22.3221**	**18.9047**	39.5318	**0.9968**	**2.0744**

**Table 4:** Statistical comparisons of multifocus image fusion on the “toys image set.”

Methods	RMSE	PFE	MAE	Entropy	SNR	PSNR	CC	ERGAS
Average method	34.2848	25.2737	19.4244	1.3784	10.7959	28.8138	0.9141	8.0940
Minimum method	19.0227	14.0230	8.5127	4.37283	15.3948	35.3721	0.9867	5.8235
DWT	12.7463	10.2732	2.0392	6.3726	20.8732	37.1203	0.9962	2.6384
SWT	12.6532	9.5487	1.1458	6.2843	20.4538	37.0410	0.9959	2.7072
DWT (Laplacian) proposed	12.6489	9.7323	1.1092	6.3743	21.8972	38.2932	0.9963	2.4832
DWT (unsharp) proposed	12.0283	9.9378	1.2872	6.4732	21.2342	38.0023	0.9962	2.6323
DWT (LF + DFT) proposed	12.0213	9.6384	0.9372	6.9983	23.2112	38.9923	**0.9969**	2.1234
SWT (Laplacian) proposed	12.4213	9.2197	0.9203	6.3283	21.8222	38.2166	0.9953	2.3003
SWT (unsharp) proposed	11.9650	9.8131	0.9288	6.3263	20.8144	37.3150	0.9959	2.9886
SWT (LF + DFT) proposed	**11.5382**	**9.2123**	**0.8812**	**7.5932**	**23.3721**	**39.3872**	0.9964	**2.0232**

**Table 5:** Statistical comparisons of multifocus image fusion on “building and card image set.”

Methods	RMSE	PFE	MAE	Entropy	SNR	PSNR	CC	ERGAS
Average method	31.3352	26.0768	18.9107	2.3554	6.0334	26.8074	0.9071	8.6514
Minimum method	17.6777	10.3879	5.4055	5.6654	14.3411	34.8047	0.9907	4.7054
DWT	12.3245	8.6483	0.0563	8.6445	18.4388	37.4885	0.9932	2.0012
SWT	11.3361	8.6096	**0.0506**	8.5664	18.8272	37.6201	0.9950	2.7695
DWT (Laplacian) proposed	10.9912	7.9874	0.0534	9.4743	20.1888	38.3732	0.9961	2.1021
DWT (unsharp) proposed	11.2323	7.9884	0.0532	9.8773	20.2981	38.1128	0.9961	2.1021
DWT (LF + DFT) proposed	9.8712	7.6653	0.0571	9.9933	21.2321	38.9901	0.9964	**1.9221**
SWT (Laplacian) proposed	10.4224	7.7726	0.0550	9.5543	9.5543	20.9489	0.9959	2.1117
SWT (unsharp) proposed	10.6771	8.3854	0.0524	9.5883	20.2085	38.2419	0.9967	2.2497
SWT (LF + DFT) proposed	**8.7712**	**7.3623**	0.0520	**10.9877**	**21.9002**	**39.2872**	**0.9972**	2.1023

The article "Hybrid Sharpening Transformation Approach for Multifocus Image Fusion Using Medical and Nonmedical Images" was published in 2021. Journal: J Healthc Eng.

**Table 6:** Statistical comparisons of multifocus image fusion on “medical images set.”

Methods	RMSE	PFE	MAE	Entropy	SNR	PSNR	CC	ERGAS
Average method	33.0091	29.2135	14.6507	1.4345	8.6566	19.9864	0.9071	11.9876
Minimum method	19.4783	9.9898	6.4475	6.5432	14.3451	31.9047	0.9801	6.4365
DWT	11.4902	9.4325	2.4554	11.2144	21.4338	32.0985	0.9833	3.0766
SWT	10.9934	9.3212	1.3554	14.5434	22.8272	38.6287	0.9951	3.7695
DWT (Laplacian) proposed	10.0120	8.0546	1.4584	13.4532	25.1645	37.3632	0.9955	3.0021
DWT (unsharp) proposed	10.2221	7.8760	1.0543	12.2233	24.2531	36.1668	0.9943	2.1981
DWT (LF + DFT) proposed	8.1100	6.5432	1.0098	14.5435	28.4334	39.9881	**0.9984**	**2.0001**
SWT (Laplacian) proposed	10.4973	6.4924	1.0730	15.7644	28.5546	35.9549	0.9981	2.5414
SWT (unsharp) proposed	9.1203	7.3432	1.0845	15.5087	27.5432	**44.4419**	0.9967	2.3297
SWT (LF + DFT) proposed	**7.1123**	**5.3332**	**1.0080**	**16.9438**	**33.4322**	43.2542	0.9982	2.1221

## Data Availability

The datasets used in this research are taken from UCI ML Learning Repository available at https://archive.ics.uci.edu/.
